# Mechanism of Action of Zhi Gan Cao Decoction for Atrial Fibrillation and Myocardial Fibrosis in a Mouse Model of Atrial Fibrillation: A Network Pharmacology-Based Study

This article has been retracted.

**DOI:** 10.1155/2022/4525873

**Published:** 2022-06-09

**Authors:** Lei Gao, Chenjing Kan, Xin Chen, Shengsong Xu, Kaihu Shi

**Affiliations:** ^1^Department of Cardiothoracic Surgery, Affiliated Hospital of Integrated Traditional Chinese and Western Medicine Nanjing University of Chinese Medicine, Nanjing, Jiangsu 210028, China; ^2^Jiangsu Province Academy of Traditional Chinese Medicine, Nanjing, Jiangsu 210028, China

## Abstract

Atrial fibrillation (AF), a commonly seen cardiac disease without optimal curative treatment option, is usually treated by traditional Chinese medicine in China. The Zhi-Gan-Cao decoction (ZGCD) is an alternative medicine for clinical use and has definitive effects. It remains to be defined regarding the specific components and related mechanisms of ZGCD for the treatment of AF. We determined the primary constituents and major targets of the herbs in ZGCD using the TCMSP, HERB, and BATMAN-TCM databases. The UniProt databank database amended and combined the prospective names to supply objective data and records. Every target connected to AF was generated using the GeneCards databank, Drugbank database, TTD, Disgenet database, and OMIM. After identifying possible common targets between ZGCD and AF, the interface network illustration “ZGCD component-AF-target” was created using Cytoscape. We obtained 175 constituents and 839 targets for seven herbal drug categories in the ZGCD and identified 1008 targets of AF. After merging and removing repetitions, 136 collective targets between the ZGCD and AF were removed using the Cytoscape system. These renowned targets were generated from 38 suitable components from among the 157 components. GO enhancement examination and KEGG enrichment analysis by Metascape identified the close connection between the critical target genes and 20 signaling pathways. Then, we injected isoproterenol subcutaneously into the mouse and gave gavage with roasted licorice soup. Two weeks later, mouse were processed and sampled for testing. The results of HE and Masson staining showed that ZGCD effectively alleviated the degree of myocardial fibrosis. As indicated by qRT-PCR and Western blotting, ZGCD significantly reduced COL1A1, COL1A2, COL3A1, and TGF-*β*1 in myocardial fibrotic tissue to reduce myocardial fibrosis and treat AF by interfering with the expression of COL1A1, COL1A2, COL3A1, and TGF-*β*1 in myocardial tissue. ZGCD may treat AF by lowering the degree of myocardial fibrosis.

## 1. Introduction

Atrial fibrillation (AF), the most persistent arrhythmia clinically found, affects approximately 33 million people across the globe [1], with one out of four middle-aged people suffering from AF in Europe and the United States [2] and 1% inflicted population in Asia [3]. The incidence of AF continues to increase directly with increase in age, and a large study conducted between 1990 and 2010 in the UK [4] reported that the AF incidence (mainly in patients older than 75 years) is related to the global AF rate. The global mortality rates have increased. AF is a global problem that endangers human life and health. Thus far, there have been many achievements with regard to AF diagnosis and treatment. However, due to complex mechanisms involved in the occurrence and development of AF, there is currently no specific optimal treatment method that can provide a clinically beneficial effect.

Specific instructions have been defined in traditional Chinese medicine (TCM) for the treatment of cardiac diseases, including arrhythmia [5]. The Zhi-Gan-Cao decoction (ZGCD), a classical formula of Chinese herbs, comprises ginger, licorice, cassia twig, ginseng, donkey-hide gelatin, *Ophiopogon japonicus*, hemp seed, Rehmannia, and jujube, among which licorice and ginseng are the most important ingredients. In China, the ZGCD has a subtle effect on arrhythmia [6]. Previous research has indicated that the activation of endothelial cells, cardiac remodeling, cardiomyocyte action potential, and platelet activation are involved in the mechanism of action of ZGCD [7–10]. A key component of ZGCD, Zhigancao, whose main components are glycyrrhizinate and glycyrrhetinic acid, plays a pivotal role in the treatment of arrhythmia [11]. Another main component, ginseng, has a definite effect on the treatment of arrhythmia [12–14].

Previous studies have shown that the ZGCD can modulate AF [8, 15], although the specific effect of ZGCD on the therapeutic targets of AF has not been explored previously. The main purpose of this study is to provide a theoretical approach that is clinically applicable to facilitate the better treatment of AF. The novelty of the current study if to focus on Chinese medicine to determine whether ZGCD can inhibit the activation of major molecular targets and signaling axis that have a connection with AF onset and progression. Accordingly, we planned to use network pharmacological systems to examine, explore, and evaluate the targets, components, and pathways involved in the multiple facets of the interactions and supervisory systems that are involved in the electrophysiology, cardiomyocyte proliferation, and apoptosis. By constructing a murine myocardial fibrosis model, we planned to evaluate whether ZGCD can treat AF by alleviating myocardial fibrosis, which could provide a basis for more intensive future research into the mechanisms of ZGCD for the disease on the one hand, and ascertain the development of novel approaches and drugs for AF treatment on the other.

## 2. Data and Methods

### 2.1. Data Preparation

The Traditional Chinese Medicine Systems Pharmacology Database and Analysis Platform (TCMSP; https://old.tcmsp-e.com/tcmsp.php) [16] was used for drug information acquisition. The main ingredients of the ZDCD, Gillian and Fresh Rehmannia root, were not found in the TCMSP. Thus, high-throughput experimental and reference-guided TCM databases HERB (http://herb.ac.cn/) [17] and BATMAN-TCM (http://bionet.ncpsb.org.cn/batman-tcm/) [18] were utilized to obtain this information. Next, the ingredients were screened by using the TCMSP. The drug targets' protein names were converted into gene names of the Human Gene Database (GeneCards; https://www.genecards.org/) [19] via the UniProt database (https://www.uniprot.org/). The enrichment analysis was performed using Metascape (https://metascape.org) [20] and using AF gene data from the GeneCards and Drug Bank (https://www.drugbank.ca/) [21].

### 2.2. Screening of Ingredients and Detection of Targets in the ZGCD

To determine the molecular drug composition of ZGCD, a systematic search of the TCMSP was performed for the title of each dynamic constituent of the ZGCD, and their chemical and structural similarities with commonly available prescription medications were compared on the US Food and Drug Administration website (https://www.fda.gov/). The pharmaceutical additives that serve therapeutic importance were evaluated using the aforementioned criteria. As the Gillian and Fresh Rehmannia root's main ingredients could not be found in the TCMSP, a high-throughput experimental and reference-guided TCM database (http://herb.ac.cn/) was used. Thereafter, the ingredients were screened by using the TCMSP.

The major ingredients of the ZGCD include licorice, ginger, cassia twig, ginseng, donkey-hide gelatin, *Ophiopogon japonicus*, and hemp seed. The chemical structure of each drug was derived after “jujube” was entered into the TCMSP database. For obtaining the structure of the drug and targets, the evaluation settings were ground on the oral bioavailability (OB; 30%) and drug-likeness (DL 0.18). Several studies have shown that testing criteria can be used to exclude unsuitable pharmaceutical ingredients [22–24]. As aforementioned, HERB (http://herb.ac.cn/) was used as the Gillian and Fresh Rehmannia root's main ingredients could not be found on the TCMSP, and the ingredients were screened by using the TCMSP.

### 2.3. Target Screening of AF

The GeneCards (HTTPS://http://www.genecards.org/) record likely delivers comprehensive and manageable statistics for all projected and annotated human genes, which are used by numerous researchers who undertake network pharmacology research [25, 26]. We used “atrial fibrillation” as the keyword to retrieve the target obtained by GeneCards in AF.

On the bioinformatics platform (https://www.bioinformatics.com.cn/) [27], the targets of ZGCD and AF were projected in a framework. Consequently, a Venn plot was constructed to obtain collective targets between herbs used in ZGCD and also to identify the shared targets of ZGCD and AF as it might be advantageous to identify the cooperative engagements of ZGCD herbal components, which would be valuable for studying the therapeutic effects of ZGCD on AF.

### 2.4. Drug Target–AF Network Building and Analysis

A medication network was built using Cytoscape software (version 3.8.2) Bisogenet [28] widget for active drug candidates via TCMSP/HERB/BATMAN-TCM as well as via the GeneCards dataset for genetic variants in glioma. Using Cytoscape, two PPI networks were constructed and validated: one for the scanned ZGCD target and one for the known AF target. The topology study gradually weeded out the central network after integrating the two systems into candidate networks.

The examination was accomplished via the CytoNCA (24) plug-in in Cytoscape to determine the following six metrics: eigen-vector centrality (EC), closeness centrality (CC), degree centrality (DC), local average connectivity (LAC), topology intermediateness (BC), and network centrality (NC). The ideal hub network was selected using the aforementioned methods.

### 2.5. Protein–Protein Interaction Network Construction

The 132 abovementioned common targets were input into The Search Tool for the Retrieval of Interacting Genes (STRING, *v*11.0, https://stringdb.org) for recovery by selecting the smallest required interconnection rating of more than two-fifths [29]; then, the PPI system of the ZGCD was evaluated for suitable components in addition to the AF-related targets.

### 2.6. Gene Ontology (GO) and Pathway-Enrichment Examination

The execution of GO and path enhancement examination of multiple items on Metascape (https://metascape.org//) were undertaken using the “Home sapiens” mode. KEGG-based enrichment pathway results were utilized for potential molecular mechanism analysis of PL@RM on AF. We used R-Studio to plot the pathways related to AF in the bubble chart.

### 2.7. Experimental Study: Drugs and Reagents

We used isoproterenol (ISO; National Medicine Standard: H50020020), purchased from Nanjing, Jiangsu, as the drug for developing the model. This model has the characteristics of high stability, easy operability, and high imitability and is currently one of the accepted methods for preparing animal models of myocardial fibrosis [30]. The ZGCD was provided by the Chinese Pharmacy of Jiangsu Hospital of Integrated Traditional Chinese and Western Medicine after ZGCD freeze-dried powder was prepared by water extraction and alcohol precipitation at the Jiangsu Provincial Hospital on Integration of Chinese and Western Medicine.

Related detection reagents, RIPA lysis buffer (P0013B), protease phosphatase inhibitor mixture (P1049), BCA protein quantification kit (P0010S), and sodium dodecyl sulphate-polyacrylamide gel electrophoresis (SDS-PAGE) loading buffer (5×; P0015L) as well as the SDSSDS-PAGE gel preparation kit (P0012A) were obtained from Beyotime (Shanghai, China). COL1A1 antibody (1 : 1000, 72026) was purchased from Proteintech (Massachusetts, USA). The COL1A2 antibody (1 : 1000, 14695-1-AP) and COL3A1 antibody (1 : 500, 22734-1-AP) were purchased from Proteintech (Chicago, USA). TGF-*β*1 (1 : 1000, ab215715) and anti-GAPDH antibodies (1 : 10000, ab8245) were supplied by Abcam (Cambridge, UK). The RNAiso Plus (9109), PrimeScript™ RT reagent Kit with gDNA Eraser (RR047A), and TB Green® Premix Ex Taq™ (RR420A) were supplied by Takara (Shiga, Japan). The design and synthesis of mouse COL1A1, COL1A2, COL3A1, TGF-*β*1, and *β*-actin primers were made by Sangong Biotech (Shanghai, China), with results presented in Table 1.

### 2.8. Animal Model

All animal experiments have gotten the approval from the Institutional Animal Care and Use Committee of Jiangsu Provincial Academy of Chinese Medicine. Healthy male specific pathogen-free C57BL/6 mice (weight: 18 ± 2 g) supplied by Shanghai Slack (production license number: SCXK (Shanghai) 2015-0002) were allowed to acclimatized to the breeding environment (temperature: 25°C, relative humidity: 45%) for 1 week and then assigned randomly into three groups: control, model, and ZGCD. The model and ZGCD groups were subcutaneously administered ISO 5 mg/kg/d to construct a mouse myocardial fibrosis model, whereas the control group received a subcutaneous injection of 1 mL/kg/d normal saline; in addition, the ZGCD group was administered 50 g/kg ZGCD daily by gavage. Two weeks later, all mice were anaesthetized with 45 mg/kg 2.5% pentobarbital sodium that was intraperitoneally injected, and blood samples were collected from the heart, stored at -80°C for 15 min of centrifugalization (3000 rpm) to obtain serum. After mouse death, the mouse's chest cavity was opened using a lateral incision, and the heart was removed. One part of the heart was placed in 4% formalin solution for hematoxylin-eosin (HE) and Masson staining, and the other part was subjected to quick liquefrozen for Wester blotting (WB) and polymerase chain reaction (PCR).

### 2.9. HE and Masson Staining

A sufficient amount of the fixed sample was placed in a 4% paraformaldehyde solution in the embedding box and then placed in an automatic dehydrator for dehydration. Following complete dehydration, paraffin embedding was performed, and the paraffinized tissue sections were obtained using a manual rotary pathological microtome. The paraffinized tissue slices were placed on an automatic slicer for baking, and 1 hour later, the slices were considered ready; some slices were put into the automatic pathological staining machine and taken out after the specified cycle was run; other slices were stained using the Masson staining kit. The slices were automatically machine-mounted, placed in a fume hood to air dry. They were taken out the next day into a slicing box for storage at indoor temperature, for the final observation and photographing under an optical microscope. We checked at least five random areas of each section and used an automated photo and image analysis system (Image-Pro Plus *v*6.0, USA) for semiquantitative evaluation.

### 2.10. qT-PCR Analysis

RNAiso Plus was used to lyse the ground mouse heart tissue, which was mixed with chloroform and then centrifuged (12000 rpm) for 15 min. After extraction, the obtained supernatant was mixed with isopropanol, followed by 10 min of centrifugalization (12,000 rpm). Following supernatant removal, 75% alcohol was used for precipitate washing. The supernatant was discarded again, and the extracted RNA was dissolved in diethyl pyrocarbonate water, followed by reverse translation into cDNA according to the Takara's reverse transcription kit instructions. Finally, the Takara fluorescent quantitative PCR kit was used to detect reverse-transcribed cDNA. When the set threshold was reached, the cycle number (CT value) of the fluorescent signal in each reaction tube was recorded. 2^−△△Ct^ was responsible for the identification of gene expression differences.

### 2.11. Western Blot Analysis

The RIPA-lysed ground mouse myocardial tissue was treated with centrifugalization (12,000 rpm, 15 min) to collect the supernatant. Protein concentration was measured with the use of the BCA protein quantification kit. Equal amount of 10 *μ*L protein samples were separated by sodium dodecyl sulfonate-polyacrylamide gel electrophoresis (SDS-PAGE) and transferred onto a polyvinylidene difluoride (PVDF) membrane (230 mA, 2.5 h) that was subjected to 1 h of cultivation with 5% bovine serum albumin solution. The PVDF membrane was then cut out according to the different molecular weights of the protein and placed in the antibody-incubation box. The diluted corresponding *Ι* antibodies were used for overnight incubation (4°C). After incubation, the corresponding II antibody was placed into the box for 2 h of indoor cultivation. ECL (Beyotime, Shanghai, China) was employed for the identification of the expression of the corresponding protein bands in the bioimager and ImageJ software (Image J Software, Bethesda, USA) for the gray value analysis of the protein band, with GAPDH as an internal reference.

### 2.12. Statistical Processing

SPSS (*v*24.0) was employed for statistical analysis. Measurement data of each group are given mean ± standard deviation ($\overset{®}{x}\pm s$). The comparison of multisample means adopts a single-factor analysis of variance. When it was in a normal distribution, the mean from pairwise comparisons was obtained using the Student's *t*-test; when the variances between groups were equal, the least-significant difference test was used; and when the variances were nonuniform, the Games–Howell test was adopted. The level of significance was *p* < 0.05.

## 3. Results

### 3.1. Herbs in the ZGCD Constituents and Its Targets

OB ≥ 30% and DL ≥ 0.18 in the TCMSP databank and a cutoff ≥ 20 in the BATMAN-TCM databank were set to monitor suitable components of cassia twig, licorice, ginger, jujube, ginseng, donkey-hide gelatin, *Ophiopogon japonicus*, fresh Rehmannia root, and hemp seed. Upon adding some significant components of the literature, 175 components were identified. The constituents of the aforementioned constituents were then typed into the UniProt databank, and these targets' information was supplemented with Swiss target prediction databank. Upon elimination of duplicates, 839 targets in the ZGCD components were obtained (Table 2).

### 3.2. Common Targets between ZGCD and AF

The keyword “atrial fibrillation” was searched in the GeneCards database, Drugbank, DTT, OMIM, and Disgenet, which returned 1008 targets after removing the duplicates.

In the bioinformatics online platform, 839 ZGCD targets and 1008 AF targets were entered, and the Venn diagram B was drawn (Figure 1). After the duplicates were removed, 157 common targets were identified between the ZGCD and AF. Furthermore, we discovered that these targets only originated from 136 active compounds, whereas the remaining 38 potential elements in ZGCD had no overlap with AF targets.

### 3.3. ZGCD-Component-AF-Target Network Analysis

In total, 36 and 157 virtual components and shared targets, respectively, between ZGCD and AF, were typed into Cytoscape 3.7.1 for the development of a visual representation in the network diagram showing the relationships between components and targets fitted to ZGCD and AF, in that order (Figure 2).

Brown represents eight herbal medicines in the ZGCD; purple, yellow, orange, and dark blue represent 136 common targets (Table 3); green, orange, pink, yellow, light cyan, purple, crimson, teal, and light red represent effective components of licorice, ginseng, jujube, *Ophiopogon japonicus*, cassia twig, hemp seed, donkey-hide gelatin, fresh Rehmannia root, and ginger, respectively (Table 4); the red line represents common effective components of different herbs. The assessment of degree shows the number of projected correlations between constituents and targets. The degree value is proportional to the importance of the component.

Subsequently, the network diagram was investigated with the use of a network analyzer. As shown in Table 3, out of 81, the top 10 constituents in ZGCD included quercetin (degree = 73), lysine (degree = 38), stigmasterol (degree = 34), kaempferol (degree = 29), luteolin (degree = 29), beta-sitosterol (degree = 20), beta-carotene (degree = 19), arachidonic acid (degree = 15), 7-methoxy-2-methyl isoflavone (degree = 14), and 1-methoxyphaseollidin (degree = 12). In Table 4, the suitable constituents of ZGCD, such as PTGS2 (degree = 111) and PTGS1 (degree = 64), displayed great action on AF medical handling through the cyclooxygenase family, which is pivotal in mediating the inflammatory reactions of AF. Moreover, ZGCD components, such as ADRB2 (degree = 47) and ADRA1B (degree = 36), strongly affected the adrenergic receptors which affected cardiomyocyte contraction. Concurrently, ZGCD affected myocardial fibrosis-related proteins, such as DPP4 [31]. The members of the collagen family related to myocardial fibrosis were also involved, such as collagen alpha-1(I) chain (COL1A1, degree = 1), collagen alpha-2(I) chain (COL1A2, degree = 1), and collagen alpha-3(I) chain (COL3A1, degree = 1). Furthermore, transforming growth factor-*β*1 (TGFB1, degree = 2), which is involved in myocardial fibrosis, is affected by ZGCD.

### 3.4. Examination of PPI Network

The abovementioned 157 common targets were entered into the STRING databank. The network interaction data of target interconnections were generated with a minimum necessary interaction score of >0.4. Each edge stands for the interplay between one protein and another. A greater degree of correlation indicated more lines and the target standing in this network (Figure 3).

### 3.5. GO Enrichment Analysis

The GO examination was executed using the Metascape data platform to clarify the mechanism that mediates the ZGCD behaviour in AF. After feeding 157 common targets to the Metascape data platform, cell components, biological process mechanism targets, and molecular functions were shown distinctly. First, the outcomes indicated an amelioration of interaction target genes to 2,365 types of biological process, which mainly regulated the response to circulation. In addition, ZGCD could regulate the response to inorganic substances in the blood, wounding, and oxygen levels. The regulation of ion transport by ZGCD is noteworthy. Additionally, the avascular process in the circulatory system and the apoptotic signaling pathway was identified.

Second, the enrichment of 149 cell constituents was focused on different cell membrane edifices, such as tissue raft, plasma membrane protein complex, contractile fibers, perinuclear cytoplasmic region, and integral components of the synaptic membrane. Moreover, the main cell constituents comprised platelet alpha granules, the external aspect of the plasma membrane, troponin complex, extracellular matrix, and the lumen of the endoplasmic reticulum.

Third, 186 molecular utility-related procedures, which mainly encompassed protein activity and receptor binding, were shown. Contrary to our expectation, ZGCD could control adrenergic receptor activity, outward rectifier potassium channel activity, cofactor binding, protein homodimerization activity, and kinase binding. On the other hand, receptor regulator activity and tetrapyrrole, protease, protein domain-specific, and troponin T binding were also important mechanisms that were shown (Figure 4).

### 3.6. Examination of KEGG Pathway Enhancement

A total of 355 KEGG pathways were identified based on 157 common targets. The 20 most essential pathways were identified using a bar plot plus a dot plot (Figure 5). The relevance of advancement was represented by *p* in the figure, and the greater the intensity of the color, the greater was the weight of the enhancement. Hypertrophic cardiomyopathy, HIF-1 (hypoxiainducible factor-1) distinguishing pathway, and adrenergic alarm signaling in cardiomyocytes were sorted, and both notable and conspicuously enhanced paths were identified that significantly contributed to the pathogenesis of myocardial fibrosis (Figures 6 and 7). Furthermore, the AGE-RAGE (advanced glycation end products and their receptor) indicative pathway is critical in diabetes, nonalcoholic fatty liver disease, tryptophan metabolism, and other metabolic pathways.

Network Analyzer was thereafter used to show the network diagram. As shown in Figure 8 and Table 5, the top 10 of the 20 KEGG pathways in ZGCD were pathways in cancer (degree = 65), proteoglycans in cancer (degree = 65), malaria (degree = 42), adrenergic alarm signaling in cardiomyocytes (degree = 41), AGE-RAGE gating pathway in diabetes-related complications (degree = 36), oxytocin-indicating path (degree = 35), Alzheimer disease (degree = 31), fluid shear stress and atherosclerosis (degree = 28), Epstein–Barr virus infection (degree = 27), and HIF-1 signaling pathway (degree = 20).

### 3.7. Pathological Changes of Mouse Myocardial Tissue

Two weeks after the mice were subcutaneously injected with ISO, the fibrous connective tissue in ISO-induced myocardial fibrosis in the model group, compared with the control group, showed significant proliferation, obvious deformation of myocardial cells, and increased collagen deposition, as indicated by the HE and Masson staining. The above-described performance was significantly reduced in the ZGCD group versus the model group (Figure 8).

### 3.8. QRT-PCT Detects the Expression of COL1A1, COL1A2, COL3A1, and TGF-*β*1 mRNA

Two weeks after modeling, the model group exhibited evidently elevated COL1A1, COL1A2, COL3A1, and TGF-*β*1 mRNA expression than the control group. While COL1A1, COL1A2, COL3A1, and TGF-*β*1 mRNA in the myocardial tissue of ZGCD-intervened mice was markedly reduced versus the model group (Figure 9).

### 3.9. Western Blotting Detects the Expression of COL1A1, COL1A2, COL3A1, and TGF-*β*1 Protein

Two weeks after modeling, the model group presented notably elevated COL1A1, COL1A2, COL3A1, and TGF-*β*1 protein expression in the myocardial tissue than the control group. While their protein levels were notably reduced in the myocardial tissue of mice in the ZGCD group versus the model group (Figure 10).

## 4. Discussion

### 4.1. Effect of ZGCD's Components on AF

136 common compounds in the ZGCD that include quercetin, stigmasterol, luteolin, kaempferol, and beta-sitosterol have good anti-inflammatory effects [32, 33]. Therefore, quercetin, stigmasterol, kaempferol, luteolin, and beta-sitosterol when used as anti-inflammatory drugs may have a good therapeutic effect on AF. Studies have reported that quercetin can modulate overactive AMPK to protect cardiomyocytes from apoptosis [34]. Cardiomyocyte apoptosis is an important factor in the remodeling of the cardiac structure during AF [35, 36]. Similarly, kaempferol, luteolin, and beta-sitosterol have antiapoptotic effects on cardiomyocytes. The fact that berberine benefits the management of AF is worth exploring. Besides, berberine has been clinically confirmed to be beneficial to AF treatment [37]. The existing studies have found that berberine inhibits AF by increasing the suitable refractory time of the atrium and elongating the atrial myocyte action potential duration [38]. Furthermore, berberine can specifically inhibit NOX isomers and directly affect ion channels to interfere with AF [39].

In addition, lysine is an essential component of the ZGCD in the treatment of AF. Studies on lysine have shown that when lysine is oxidised by lysine oxidase, it will cause interconnecting linkages among the lysine residues of lysine-rich proteins. Changes in the expression of lysine oxidase occur in numerous heart diseases and are considered the key aspects that mediate fibrosis in related tissues, including those in AF [40]. However, other studies on lysine and AF have not been reported.

PTGS2 and PTGS1 belonging to cyclooxygenase are essential targets of atrial fibrillation. PTGS1 can promote platelet aggregation, and it can inhibit effectively anticoagulant, thereby playing the role of treating atrial fibrillation [41]. PTGS1 can induce the production of PTGS2, and PTGS2 is a critical link in triggering the subsequent inflammatory response. PTGS2 inhibitors have been used clinically. That is, nonsteroidal anti-inflammatory drugs can induce AF when treating related diseases [42]. It shows that ZGCD can interfere with atrial fibrillation by regulating PTGS2 and PTGS1.

In summary, among the 136 active ingredients in the ZGCD, the intervention for AF mainly focuses on improving myocardial inflammation, apoptosis, and cardiac ion channels. However, most of the ingredients are currently not studied directly in the treatment of AF.

### 4.2. Myocardial Fibrosis-Related Protein in AF

Notably, related proteins involved in myocardial fibrosis are essential in AF treatment with ZGCD. These include COL1A1, COL1A2, and COL3A1 in the collagen family, and TGF-*β*1, which is an essential protein that mediates fibrosis. In the GO KEGG results, TGF-*β*1 in the cardiac hypertrophy pathway was closely related to AF.

The development and manifestation of AF is associated with structural, electrical, and metabolic remodeling, which plays a fundamental part, and the key to the maintenance and recurrence of AF is atrial remodeling [43]. Atrial fibrosis is the primary pathological manifestation and sign of atrial structural remodeling, and the severity of AF increases proportionally with the degree of atrial fibrosis, which tends to become permanent [44]. Myocardial fibrosis will further cause myocardial hypertrophy [45]. Cardiac fibrosis, which is the pathological basis of AF, comprises various injury factors that cause abnormal collagen fiber deposition in the interstitium of cardiomyocytes. However, the pathogenesis of AF-related myocardial fibrosis remains unclear. Therefore, based on the pathogenetic role of myocardial fibrosis in AF, blocking and inhibiting myocardial fibrosis is an essential measure in the clinical treatment of AF.

In subsequent experiments in mice, it was observed that ZGCD can significantly improve the degree of fibrosis and collagen deposition in mouse myocardial tissue. From the results of qRT-PCR and Western blotting detection, it can be seen that ZGCD can reduce the expression of COL1A1, COL1A2, and COL3A1 genes and proteins in the fibrotic pathway of mice with myocardial fibrosis. ZGCD has the same effect on TGF-*β*1 in the cardiac hypertrophy pathway. This is consistent with the results obtained from the network pharmacology analysis. Cardiac fibrosis is a myocardial scarring event featured in increased type I collagen deposition, as well as cardiac fibroblast activation and differentiation into myofibroblasts [46]. The main process involves damage to cardiomyocytes, including apoptosis, autophagy, oxidative stress, and inflammation [47, 48], and to the corresponding slave cardiomyocytes (CMS), endothelial cells, immune cells, macrophages, etc. [49]. During this process, CMS rapidly undergo apoptosis, and endothelial cells regulate the inflammatory response. Furthermore, the proliferating immune cells infiltrate the damaged myocardium to clear away the necrotic tissue and release various growth factors and cytokines like connective tissue growth factor and TGF-*β* [50, 51]. In response to these cytokines, cardiac fibroblasts are activated and activate extracellular matrix- (ECM-) producing cells in myocardial tissue. The cells producing the myocardial ECM are various myocardial interstitial cells [52–54], which can produce various collagen fibers in myocardial tissue. In the adult myocardium, the main components of myocardial tissue are type I collagen fibers (~85%) and type III collagen fibers (~11%), and the rest collagen fibers have types IV, V, VI, and other fibers [55]. When collagen deposits increase, the ratio and arrangement of various types of collagen will lead to myocardial fibrosis, which induces the release of more inflammatory factors, which further aggravates the process of fibrosis [56].

It can be seen that COL1A1, COL1A2, COL3A1, and TGF-*β*1, which are involved in stimulating the activation of cardiac fibroblasts, are essential in treating of myocardial fibrosis using ZGCD for AF.

However, some limitations still exist in this study. Despite effectual components and quotidian target genes in the ZGCD and AF interactions have been identified through network pharmacology, the target gene has not been further identified to obtain key genes. Besides, the treatment effect of ZGCD on atrial fibrillation has not been fully investigated; was intervening myocardial fibrosis the only therapeutic mechanism for ZGCD on atrial fibrillation? Well-designed *in vitro* and *in vivo* experiments are needed in the follow-up study.

## 5. Conclusions

In conclusion, network pharmacology identified effectual components (81) and quotidian target genes (157) in the ZGCD and AF interactions. According to the PPI system, GO enhancement evaluation, and KEGG track enhancement evaluation, ZGCD may treat AF by lowering the degree of myocardial fibrosis. Finally, experiments in mice further demonstrated the therapeutic effect of ZGCD on myocardial fibrosis. The prospect of this study is to provide new therapeutic options for patients with atrial fibrillation.

## Figures and Tables

**Figure 1:** Target matching is presented in Venn diagram to illustrate the overlap between the ZGCD and AF targets. Targets of herbs in the ZGCD are represented in red, and the targets of AF are shown in green.

**Figure 2:** The network drawing for the interaction of the ZGCD-component-AF target.

**Figure 3:** (a) The protein–protein interaction (PPI) system; (b): PPI network targets (top 30).

**Figure 4:** GO analysis. Natural procedures, cellular constituents, and molecular functions are examples of molecular functions. (a) Barplot BP, (b) Dotplot BP, (c) Barplot CC, (d) Dotplot CC, (e) Barplot MF, and (f) Dotplot MF (*p* 0.05). BP: biological process; CC: cellular component; MF: molecular function.

**Figure 5:** The examination of the KEGG pathway enhancement in AF diagnosed with ZGCD. ZGCD: Zhi-Gan-Cao decoction; AF: atrial fibrillation.

**Figure 6:** Hypertrophic cardiomyopathy identified by the examination of KEGG pathway enhancement.

**Figure 7:** Network diagram of the interaction of the ZGCD–KEGG pathway–AF target.

**Figure 8:** Pathological changes of myocardial fibrosis induced by isoproterenol: (a) paraffinized cardiac tissue slices stained with hematoxylin and eosin (HE, 100x); (b) slices stained with Masson's trichrome (100x). ^∗^*p* < 0.05 vs. control, ^#^*p* < 0.05 vs. model.

**Figure 9:** QRT-PCR detects the mRNA expression of genes related to myocardial fibrosis in mice. (a) mRNA expression of COL1A1. (b) mRNA expression of COL1A2. (c) mRNA of COL3A1. (d) mRNA expression of TGF-*β*1.

**Figure 10:** Western blotting was used to detect the expression of myocardial fibrosis protein in mice. (a) Western blotting was used to detect the expression of COL1A1, COL1A2, COL3A1, and TGF-*β*1 protein. (b) Statistical diagram of Western blotting results. ^∗^*p* < 0.05 vs. control, ^#^*p* < 0.05 vs. model.

**Table 1:** The primer sequence of COL1A1, COL1A2, COL3A1, TGF-*β*1, and *β*-actin.

Gene		Primer sequence
COL1A1	Forward	5′TGAACGTGGTGTACAAGGTC3′
	Reverse	5′CCATCTTTACCAGGAGAACCAT′3

COL1A2	Forward	5′GCCTAGCAACATGCCAATATTT3′
	Reverse	5′GAATACTGAGCAGCAAAGTTCC′3

COL3A1	Forward	5′GAAAGAATGGGGAGACTGGAC3′
	Reverse	5′TACCAGGTATGCCTTGTAATCC3′

TGF-*β*1	Forward	5′CCAGATCCTGTCCAAACTAAGG3′
	Reverse	5′CTCTTTAGCATAGTAGTCCGCT′3

*β*-Actin	Forward	5′CTACCTCATGAAGATCCTGACC′
	Reverse	5′CACAGCTTCTCTTTGATGTCAC′3

**Table 2:** The constituents' number and targets projected with regard to the herbs in the ZGCD.

Herbs	Components number	Predicted targets number
Liquorice	92	235
Fresh Rehmannia root	6	44
Ginseng	22	118
Jujube	29	211
Donkey-hide gelatin	3	400
*Ophiopogon japonicus*	18	243
Hemp seed	6	114
Ginger	5	57
Cassia twig	11	66

**Table 3:** The top 10 effective constituents of herbs in ZGCD.

Number	Degree	Constituents	Liquorice		Ginseng	Jujube	Donkey-hide gelatin	*Ophiopogon japonicus*	Hemp seed	Ginger	Cassia twig
1	73	Quercetin	√			√					
2	38	Lysine					√				
3	34	Stigmasterol		√	√	√		√	√	√	
4	29	Kaempferol	√		√						
5	29	Luteolin							√		
6	20	Beta-sitosterol		√	√	√				√	√
7	19	Beta-carotene				√					
8	15	Arachidonic acid							√		
9	14	7-Methoxy-2-methyl isoflavone	√								
10	12	1-Methoxyphaseollidin	√								

ZGCD: Zhi-Gan-Cao decoction; AF: atrial fibrillation.

**Table 4:** The targets between ZGCD and AF (157).

Number	Degree	Name	Number	Degree	Name	Number	Degree	Name
1	111	PTGS2	54	2	CD40LG	107	1	GAA
2	70	PPARG	55	2	CDKN1A	108	1	GJA5
3	67	NOS2	56	2	CYP1A1	109	1	HADHA
4	64	PTGS1	57	2	EGFR	110	1	HSPA5
5	61	SCN5A	58	2	F3	111	1	HSPB1
6	58	F10	59	2	GJA1	112	1	HTT
7	47	ADRB2	60	2	HIF1A	113	1	IGF1
8	38	DPP4	61	2	IL10	114	1	IKBKB
9	31	ADRA1B	62	2	IL2	115	1	KCNA2
10	26	ACHE	63	2	IL6	116	1	KCNA3
11	22	F7	64	2	LEP	117	1	KCNA5
12	21	KCNH2	65	2	MMP9	118	1	KCNC1
13	16	NOS3	66	2	MTR	119	1	KCND2
14	14	ADRA1D	67	2	MYC	120	1	KCND3
15	10	MAOB	68	2	PLAT	121	1	KCNE5
16	8	ADRA1A	69	2	PON1	122	1	KCNIP2
17	8	CASP3	70	2	PPARA	123	1	KCNK2
18	7	AKT1	71	2	RNASE1	124	1	KCNQ1
19	7	NR3C2	72	2	RNF207	125	1	MAOA
20	6	BCL2	73	2	RYR3	126	1	MAP2K4
21	6	CHRM2	74	2	SELE	127	1	MMP3
22	6	DRD2	75	2	STAT1	128	1	MYBPC3
23	5	MAPK1	76	2	TGFB1	129	1	NFE2L2
24	5	XDH	77	2	TP53	130	1	NKX2-1
25	4	CASP9	78	2	VCAM1	131	1	NPPA
26	4	CAT	79	2	VKORC1	132	1	PCNA
27	4	CCND1	80	1	ABCA1	133	1	PECAM1
28	4	CYP3A4	81	1	ADRA2A	134	1	PLG
29	4	HMOX1	82	1	ADRB1	135	1	POLG
30	4	ICAM1	83	1	AGXT2	136	1	PRODH
31	4	IL1B	84	1	ALB	137	1	RAF1
32	4	MMP1	85	1	APOE	138	1	SCN10A
33	4	NR1I2	86	1	APP	139	1	SELP
34	4	PRKCA	87	1	ATP1A2	140	1	SERPINE1
35	4	TNF	88	1	AVP	141	1	SLC19A2
36	3	ADORA1	89	1	CACNA1D	142	1	SLC22A6
37	3	ADRA2B	90	1	CACNA1S	143	1	SLC25A4
38	3	CASP8	91	1	CACNA2D1	144	1	SOD2
39	3	CETP	92	1	CASP1	145	1	SPP1
40	3	CYP1A2	93	1	CCL2	146	1	TERT
41	3	IFNG	94	1	COL1A1	147	1	TFAP2B
42	3	MMP2	95	1	COL1A2	148	1	TH
43	3	NFKBIA	96	1	COL3A1	149	1	THBD
44	3	SOD1	97	1	CRP	150	1	TLR4
45	3	VEGFA	98	1	CTNNB1	151	1	TNFRSF1A
46	2	ADRA2C	99	1	CXCL8	152	1	TNNC1
47	2	ANK3	100	1	CYP2B6	153	1	TNNI2
48	2	APOB	101	1	CYP2E1	154	1	TNNI3
49	2	APOH	102	1	DLD	155	1	TNNI3K
50	2	APRT	103	1	EDN1	156	1	TNNT1
51	2	CAV1	104	1	FAS	157	1	TNNT2
52	2	CAV3	105	1	FOS			
53	2	CD36	106	1	FXN			

ZGCD: Zhi-Gan-Cao decoction; AF: atrial fibrillation.

**Table 5:** 157 KEGG pathways between ZGCD and AF.

No.	Degree	Name
1	65	Pathways in cancer
2	65	Proteoglycans in cancer
3	42	Malaria
4	41	Adrenergic signaling in cardiomyocytes
5	36	AGE-RAGE signaling pathway in diabetic complications
6	35	Oxytocin signaling pathway
7	31	Alzheimer disease
8	28	Fluid shear stress and atherosclerosis
9	27	Epstein–Barr virus infection
10	20	HIF-1 signaling pathway
11	20	Nonalcoholic fatty liver disease
12	19	Hypertrophic cardiomyopathy
13	14	Huntington disease
14	12	Thyroid cancer
15	10	Epithelial cell signaling in *Helicobacter pylori* infection
16	10	Transcriptional misregulation in cancer
17	10	Longevity-regulating pathway
18	8	Allograft rejection
19	8	Tryptophan metabolism
20	7	Complement and coagulation cascades

## Data Availability

The data used to support the findings of this study are available from the corresponding author upon request.
